# Surgical Selection of T1 Stage Renal Tumor Resection Based on Imaging MAP Score under Smart Medical Care

This article has been retracted.

**DOI:** 10.1155/2022/1947504

**Published:** 2022-05-18

**Authors:** Hongtao Zong, Qiang Xia, Liansheng Zhang, Jin Zhu

**Affiliations:** ^1^Department of Urology, Wuxi No. 9 People's Hospital Affiliated to Soochow University, Wuxi 214062, Jiangsu, China; ^2^Department of Urology, the Second Affiliated Hospital of Soochow University, Suzhou 215004, Jiangsu, China

## Abstract

Smart medical uses the medical information platform and the current technological means to enable the process of sharing information between medical staff and medical equipment. The combination of current technology and the medical field has become the norm. In the future, more artificial intelligence technologies will be integrated into the medical field to promote the development of medical care. At present, the information on the Internet is very large and complex, and general search engines often do not have knowledge in certain professional fields and can only perform shallow keyword searches. Therefore, it is difficult to meet people's medical diagnosis needs, and smart medical care can solve these needs. Medical imaging refers to the technology or process of obtaining internal tissue images of a certain part of the human body for medical research, including medical imaging systems and medical image processing. Medical image processing refers to the further processing of the obtained images, the purpose of which is either to restore the original image that was not clear enough or to highlight some characteristic information in the image. The purpose of this paper is to study the research on the selection of T1 stage renal tumor resection based on the imaging MAP score under smart medical care. It is hoped that through smart medicine and medical imaging technology, it can help renal tumor resection, reduce the sequelae of renal tumor resection, and promote the development of medical services. This paper proposes applying natural language processing technology to the medical field, creating an intelligent diagnosis assistance system, and using the existing medical record data to realize the corresponding medical assistance functions. It studies the class imbalance problem prevalent in medical datasets and provides better solutions through ensemble learning techniques to improve classifier performance when the number of positive and negative samples is unbalanced. The experimental results in this paper show that the creatinine of patients undergoing renal tumor resection combined with smart medicine and imaging technology is stable at 75 mol/L, while the creatinine is stable at 71 mol/L in other methods. It shows that the postoperative effect of smart medical treatment and imaging technology is better.

## 1. Introduction

With the development of the economy, people's living standards begin to improve, people pay more and more attention to people's health, and the medical demand begins to increase, resulting in a shortage of medical resources in the society and a shortage of medical staff. How to optimize the allocation of resources on the basis of limited medical resources, improve the utilization rate of medical resources, and alleviate the contradiction between doctors and patients is an urgent problem to be solved at present. The conflict between doctors and patients may be caused by the lack of smooth channels for rights protection or the accident caused by the patient's own reasons. Smart medical care can meet various medical needs through intelligent methods, provide patients with convenient and humanized services, alleviate medical conflicts, and obtain effective health services. Tumor is a deadly disease that threatens human health. According to survey data, there are more than 1,000 new cases of cancer every year in the world, and nearly half of them die from tumors, and the incidence group is getting younger and younger. At present, there is no specific epidemiological data on tumor research, but all tumor patients should receive diagnosis and treatment as soon as possible, control the progression of the disease, and avoid serious damage to the body as much as possible. Tumors can be divided into malignant tumors, benign tumors, borderline tumors, and cancerous tumors according to the tumor type. In order to improve the success rate of renal tumor resection, this paper combines renal tumor resection with smart medical care to reduce the probability of postoperative complications and promote the development of medical care.

The use of smart medical systems to integrate cases can realize the medical auxiliary role of cases, improve the efficiency and effectiveness of diagnosis, promote the scientificization of clinical medical treatment, and avoid diagnosis accidents caused by personal mistakes of medical staff. Combining smart medicine and medical imaging technology with renal tumor resection can improve the success rate of surgery, reduce surgical complications, and promote the development of medical care to a certain extent.

For the first time, this paper proposes standardizing the business process in the intelligent medical environment, simulating the randomness of the environment and the concurrency of the process after the introduction of intelligent medical equipment and systems, and improving the efficiency in the actual work process. This article not only evaluates the intraoperative and postoperative outcomes but also monitors the long-term postoperative renal outcomes for a comprehensive understanding. According to the instrument characteristics of the microscopic hyperspectral imaging system, the optimal data preprocessing and visualization scheme was proposed, which provided data support for pathological analysis. Microscopic hyperspectral imaging systems provide spectral and spatial information in the visible, near-infrared, and short-wave infrared ranges for multiplexing and biological detection, with stable and unique narrow pulses.

## 2. Related Work

As a social subject, “people” also pay the most attention to people. The current living conditions are improving day by day, and people are paying more and more attention to health, which leads to a shortage of medical resources. How to alleviate the contradiction of medical resources is the current hot spot. With the development of the Internet of Things, information sharing among various smart devices around the world has become easy. In such an environment, smart healthcare also needs to be accelerated to provide a remote diagnosis to patients around the world. However, since sensitive information about patients is disseminated using open channels, namely, the Internet, there is a potential for misuse of this information. Chaudhary R proposes a novel lattice-based secure cryptosystem for Smart Healthcare in Future Smart Cities (LSCSH). LSCSH uses a lightweight key exchange and authentication mechanism in several stages. The proposed scheme has been evaluated in terms of communication and computational cost compared to other schemes, and the results show that the system handles smart medical data securely [1]. Alhamid M F proposes a breast cancer monitoring system to be used as part of smart healthcare. Breast cancer is one of the major causes of death in young and old women, yet women are often reluctant to see a doctor due to social and psychological barriers. Smart cloud-based solutions can help women overcome this barrier. In the proposed system, mammograms can be taken from a machine and processed and analyzed in the cloud. In the system, the authors use local binary patterns (LBPs) and cooccurrence matrices of regions of interest from mammographic images. Experimental results show that the proposed system can achieve more than 98% accuracy in distinguishing between normal and mass and more than 87% accuracy in distinguishing benign from malignant [2]. The user identification aspect of smart medical systems is considered very promising. But improving the authentication accuracy is a big challenge, especially for scenarios with a large number of users. Therefore, Zhang Y proposed a parallel ECG-based authentication called PEA. The authors propose a hybrid ECG feature extraction method that fuses benchmark-based and nonbenchmark-based features to extract more comprehensive ECG features, thereby improving authentication stability. Furthermore, the authors propose a parallel ECG pattern recognition framework to improve the recognition efficiency in multiple ECG feature spaces. Through experiments, the performance of the proposed authentication is verified [3]. Since health is a sensitive issue, it should be treated with utmost safety and caution. Ghoneim A proposes a new medical image forgery detection system for the healthcare framework to verify that healthcare-related images have not been altered. The system processes the noise map of the image, applies a multiresolution regression filter on the noise map, and provides the output to support vector machine-based and extreme learning-based classifiers. Noise maps are created in edge computing resources, while filtering and classification are done in core cloud computing resources. In this way, the system can work seamlessly in real time. The bandwidth requirements of the proposed system are also reasonable [4]. Deep convolutional neural network methods have difficulty analyzing specific regions of an image and the relationships between those regions. Xie Y proposed an image aesthetic quality assessment method based on the complementary combination of deep features and handcrafted features. He selected and designed five sets of aesthetically relevant handcrafted features, including line and angle features and sharpness comparison features. Deep features are obtained using the Siamese network. A support vector regression algorithm is then applied to evaluate the image aesthetic quality score based on those handcrafted and deep features. Experimental results show that the proposed method outperforms existing methods, and the results are consistent with subjective evaluation results [5]. Tuberous sclerosis complex (TSC) is an inherited tumor syndrome caused by mutations in TSC1 or TSC2 that lead to abnormal activation of mTOR. In this study, Narov K examined the efficacy of GSK2126458 with rapamycin in the treatment of kidney tumors in genetically engineered Tsc2 ± mice. He found that both GSK2126458 and rapamycin resulted in a significant reduction in the number and size of solid kidney tumors. GSK2126458 also significantly reduced the number and size of all lesions, albeit to a lesser extent compared to rapamycin. In addition, GSK2126458 and rapamycin inhibited tumor cell proliferation. Importantly, GSK2126458 increased apoptosis in solid tumors, whereas rapamycin did not [6]. Extreme learning machines (ELMs) have recently attracted increasing attention in pattern recognition and machine learning fields due to their simplicity, speed, and good generalization ability. To study the performance of ELM on hyperspectral images (HSI), Zhou Y proposed two spatial-spectral composite kernel (CK) ELM classification methods. In the proposed CK framework, a single spatial or spectral kernel consists of an activation function-based kernel and a general Gaussian kernel, respectively. The proposed method inherits the advantages of ELM and has an analytical solution that directly implements multiclass classification. Experimental results on three benchmark hyperspectral datasets show that the proposed ELM with CK method outperforms general ELM, SVM, and SVM with CK method [7]. Obtaining hyperspectral images (HSIs) with the high spatial resolution is challenging due to the limitations of existing imaging hardware. Superresolution (SR) focuses on methods to improve spatial resolution. Li Y proposes an HSI SR method by combining the Spatial Constraint (SCT) strategy with the Deep Spectral Disparity Convolutional Neural Network (SDCNN) model. It superresolves HSI while preserving spectral information. The SCT strategy constrains the low-resolution (LR) HSI generated by the reconstructed high-resolution (HR) HSI to be spatially close to the input LR HSI [8]. Although these theories have discussed renal tumor resection to a certain extent, they are less integrated with smart medicine and are not practical.

## 3. Methods for the Selection of T1 Stage Renal Tumor Resection Based on Imaging MAP Score under Smart Medical Care

### 3.1. Smart Healthcare

The United States' plan for smart medical technology was launched at the beginning of the last century, and it was also the earliest research on smart medical technology [9]. Due to its remarkable achievements in the medical field, Europe and Japan also launched discussions on intelligent medical technology. This technology was first applied to large hospitals, where doctors use intelligent medical instruments to detect the vital signs of patients to relieve medical pressure [10, 11]. Smart medical care refers to meeting the various needs of users in daily medical treatment in an intelligent way and providing users with convenient, fast, and humanized medical services through technologies such as the Internet of Things, big data, and cloud computing. With the continuous development and progress of science and technology, Internet technology has begun to be practical in the medical neighborhood, and smart medical technology is also constantly improving, showing a trend of portability, making it possible to provide personalized services for family members [12, 13]. It provides users with medical services such as online medical treatment, appointment registration, electronic medical records, and postdiagnosis tracking.  Figure 1 shows the structure of the smart medical system.

American companies were the first to develop a wearable telemedicine monitoring system. The patient wears the device on the body, the device can detect the human body's ECG signal, and the patient can observe their own ECG signal through the device [14, 15]. The device stores the collected data and location information in the computer, analyzes and processes the data through special software, and finally forms a data analysis diagram for reference [16]. One of them is a smart wearable device that can detect the motion state of human joints and can remotely monitor and monitor patients who have undergone joint surgery. In this way, the process of going to the hospital can be avoided, and the patient can complete the rehabilitation treatment at home, saving the medical resources of the hospital and the treatment cost of the patient [17]. There is also a ring sensor that patients can wear on their wrists to monitor the patient's pulse. The device also has an alarm algorithm set up to keep the wristband and the patient under monitoring at the same time [18, 19].  Figure 2 shows the early smart medical structure.

Compared with the research process of Western countries, China's research on smart medical technology started late, and the research depth cannot be compared with it [20]. China's exploration of smart medical care lies in the design of the hospital service environment and service process, the behavioral psychology of patients seeking medical treatment, their attitude towards mobile medical care, and the advantages of mobile medical treatment. It was not until the early 1990s that the application of smart medical care appeared; that is, the PLA General Hospital conducted a joint consultation with a foreign hospital through remote video [21, 22]. But until now, the technology has not been widely used in China. Traditional institutional obstacles make it difficult to share information in the medical industry and hinder the construction of a basic network for the development of the Internet of Things; China's smart medical products and technical standards are not perfect, and there is a phenomenon of applying nonprofessional standards. A university has developed a small nurse system consisting of a home monitor and a hospital server, which successfully enables patients to monitor ECG and blood pressure at home, and can analyze the data in real time. If the system thinks that the data is abnormal, it will send the abnormal data to the server of the hospital, and then experts will check the abnormal data and organize consultation [23, 24].  Figure 3 shows the specific working structure.

In addition, the Academy of Military Medical Sciences has developed a wearable medical monitoring system, which distributes information-gathering instruments on the coat. If I want to perform detection, it can be directly put on the coat [25, 26]. The information collected by the device can be transmitted to the electronic device through the wireless network, which is convenient for medical staff to view [27]. The system can realize remote monitoring and mobile monitoring at the same time [28]. With the development of Internet technology, smart medical systems have gradually attracted the attention of Chinese people. At present, smart medical-related systems have been used in the market. Using the Internet of Things technology, we monitor the daily life of the guardian and detect various vital signs of the human body. If the patient walks out of the monitoring range or has an accident, the system will notify the nearest hospital and family members to provide timely assistance to the ward, which greatly improves the cure rate [29, 30].  Figure 4 shows the structure of the smart medical system.

### 3.2. Image Processing

Medical imaging is indispensable in modern medical care; especially in the surgical process, imaging technology plays a pivotal role. The subject of this study is the relationship between renal tumor resection and medical imaging, so it is necessary to focus on image processing techniques.

Entropy was originally used to represent the energy distribution in thermodynamics. In recent years, it has also achieved certain development in the medical field. We define its function expression as

(1) $$\begin{array}{c} F\left(a\right)=-q\sum_{i=1}^{m}k_{i},\;\ln\left(k_{i}\right). \end{array}$$

Among them, when ∑_*i*=1_^*m*^*k*_*i*_=1, *k*1=*k*2=*k*3=⋯*km*, *F* takes the maximum value.

(2) $$\begin{array}{c} Q\left(a\right)=\int_{0}^{1}\left(Q_{\mathrm{int}}\left(a\right)+Q_{\text{image}}\left(a\right)\right)\text{d}c, \end{array}$$

where *Q*_int_(*a*) represents the internal energy, and its form is as follows:

(3) $$\begin{array}{c} Q_{\mathrm{int}}\left(a\right)=\frac{1}{4}\left(\chi \left(c\right){\left|a^{\prime }\left(c\right)\right|}^{3}+\eta \left(c\right){\left|a^{\prime \prime }\left(c\right)\right|}^{3}\right). \end{array}$$

Among them, *χ*(*c*) and *η*(*c*) represent the weight coefficient.

In the actual processing of the image, the gray value of the image fluctuates very obviously in a small range. In order to find the peak value accurately, the gray image of the image needs to be intervened. Grayscale images only need one byte per pixel to store the grayscale value. Grayscale images are usually obtained by measuring the brightness of each pixel in a single electromagnetic spectrum (such as visible light), so grayscale images can avoid banding distortion. We use the exponential smoothing method for smoothing, and its function expression is as follows:

(4) $$\begin{array}{c} Y\left(a\right)=\left(1-\beta \right)*Y\left(q-1\right)+\beta *H\left(a\right), \end{array}$$

where *a* represents the gray value, *q*−1 represents the smoothed value, *H*(*a*) represents the original value, and *β* represents the constant.

Smoothing an image is a very common technique. The pixel points are used to calculate the weighted average value to calculate the gray value. The weighted average value is its core content. Image smoothing refers to the presence of certain areas of the image that vary greatly in brightness due to factors such as the sensor and the atmosphere. In order to suppress noise, the processing method to flatten the image brightness is image smoothing.

(5) $$\begin{array}{c} y\left(a\right)=\frac{u}{\partial \sqrt{2\pi }}e^{-{\left(a-\varepsilon \right)}^{2}/2\partial^{2}}. \end{array}$$

Among them, the expected value of the Gaussian distribution is *ε*, the standard deviation is *∂*, and the standard Gaussian distribution is *ε* = 0, *∂*  = 1.

In practical processing, we often use Gaussian blurred two-dimensional Gaussian distribution density distribution function, and its expression is expressed as

(6) $$\begin{array}{c} H\left(a,b\right)=\frac{1}{2\pi \lambda^{2}}e^{-a^{2}+b^{2}/2\lambda^{2}}, \end{array}$$

where *λ* represents the standard deviation.

In information theory, entropy can effectively reflect the information contained in the event, so in specific use, the change of the entropy value of the image can be used for target segmentation. Since the texture of the background image is relatively fixed, this shows that its entropy value is relatively determined [13]. Its mathematical expression is as follows:

(7) $$\begin{array}{c} T_{t}=-\sum_{a=1}^{X}\sum_{b=1}^{Y}R_{ab}\log\;R_{ab},\\ R_{ab}=\frac{w\left(a，b\right)}{\sum_{a=1}^{X}\sum_{b=1}^{Y}w\left(a，b\right)}, \end{array}$$

where *w*(*a*, *b*) is the gray value of the pixel in the image, and *x* and *y* are the image size.

Because the logarithmic operation is used to calculate the local entropy of the image, the calculation amount is large and the speed is slow. Then, when *R*_*ab*_ ≪ 1, using the Tepler to remove the high-order terms, we can obtain

(8) $$\begin{array}{c} T_{t}\approx -\sum_{a=1}^{X}\sum_{b=1}^{Y}R_{ab}\left(R_{ab}-1\right)=1-\sum_{\left(a，b\right)\varepsilon \left(X,Y\right)}R_{ab}^{2}. \end{array}$$

When the pixels in the image change slowly, an image gray value composed of *U* pixels can be expressed as

(9) $$\begin{array}{c} p=\frac{1}{U}\sum_{i}g\left(a，b\right), \end{array}$$

where *u* represents the image composed of pixels.

(10) $$\begin{array}{c} \frac{\delta a\left(z,x\right)}{\delta x}=W=\eta \left(z,x\right)\bar{X}+\kappa \left(z,x\right)\bar{Y}, \end{array}$$

where formula (10) represents the curve evolution theory, and *W* represents the velocity vector of the curve.  Figure 5 is a schematic diagram of the evolution direction of the curve.


(11) $$\begin{array}{c} \bar{X}=\frac{\left(-\varphi_{k},2\right)}{\sqrt{2+\varphi_{k}^{3}}}, \end{array}$$

(12) $$\begin{array}{c} \bar{Y}=\frac{\left(2,\varphi_{k}\right)}{\sqrt{2+\varphi_{k}^{3}}}. \end{array}$$

Formula (11) and formula (12) represent the normal vector and the tangential vector.

(13) $$\begin{array}{c} R\left(a\right)=\left[\left(h,j\right),p\left(h,j,a\right)=r\right]. \end{array}$$

Among them, *p*(*h*, *j*, *a*) represents the time-varying level set, and *R*(*a*) represents the evolution curve point set.

(14) $$\begin{array}{c} \frac{\text{d}p}{\text{d}a}=\frac{\alpha p}{\alpha a}+\nabla p*\frac{\alpha \left(f,g\right)}{\alpha a}=0, \end{array}$$

(15) $$\begin{array}{c} \frac{\alpha \left(f,g\right)}{\alpha a}=\frac{\alpha i}{\alpha a}=\overset{⟶}{W}. \end{array}$$

Formula (14) and formula (15) represent the total derivative of formula (13).

(16) $$\begin{array}{c} \frac{\alpha p}{\alpha a}=-\nabla p*\overset{⟶}{W}\\ =-\left|\nabla p\right|\overset{⟶}{Y}*\overset{⟶}{W}. \end{array}$$

Among them, $\overset{⟶}{W}$ represents the evolution speed of the level set, and $\overset{⟶}{Y}$ represents the normal component of the level set evolution, as shown in Figure 6.


(17) $$\begin{array}{c} T\left(a\right)=\int_{0}^{1}G\left(b,c,c_{b}\right)\text{d}b. \end{array}$$

Formula (17) is a variational function expression.

(18) $$\begin{array}{c} T\left(c+o\right)=T\left(c\right)+\int_{0}^{1}\left(o\frac{\alpha G}{\alpha c}-o\frac{\text{d}}{\text{d}c}\left(\frac{\alpha G}{\alpha c^{\prime }}\right)\right)\text{d}c,\\ \frac{\alpha G}{\alpha c}-\frac{\text{d}}{\text{d}c}\left(\frac{\alpha G}{\alpha c^{\prime }}\right)=0. \end{array}$$

When the value of *T*(*c*) is very small, the value of *T*(*c*+*o*) can be seen as constant.

## 4. Experiment on the Selection of T1 Stage Renal Tumor Resection Based on Imaging MAP Score under Smart Medical Care

### 4.1. Experimental Subjects

In this experiment, in order to explore the clinical situation of renal tumor resection, we surveyed the patients who underwent renal tumor resection within a certain period of time in city A. Among the subjects under investigation, only had renal tumor disease, avoiding the influence of other etiologies on the experiment.

According to the data in Table 1, 148 patients were investigated in this experiment, including 83 male patients and 65 female patients. From the perspective of the composition of male and female patients, male patients accounted for 56.1%, and female patients accounted for 43.9%. The proportion of male patients with renal tumors was slightly higher than that of female patients. 3 patients were 0–20 years old, 30 patients were 21–40 years old, 44 patients were 41–60 years old, and 71 patients were 60–80 years old. According to the age of onset, the prevalence of renal tumors increases with age, especially in people over 60 years old.

According to the data in Table 2, in this experiment, we divided the patients into three groups, and the three groups of patients were all renal tumor patients, excluding the interference of other conditions on the surgical results. The first group consisted of 19 patients, 9 of whom opted for open surgery. There were 20 patients who chose laparoscopic surgery, 7 patients who chose simple laparoscopic surgery, and 13 patients who chose imaging laparoscopic surgery. There are 60 patients in the second group, 25 patients choose open surgery, 35 patients choose laparoscopic surgery, 25 patients choose simple laparoscopic surgery, and 10 patients chose imaging laparoscopic surgery. There are 40 patients in the third group, 32 patients choose open surgery, 8 patients choose laparoscopic surgery, 5 patients choose simple laparoscopic surgery, and 3 patients choose imaging laparoscopic surgery. According to the survey data, more patients choose laparoscopic surgery, and fewer patients choose other methods for surgery.

### 4.2. Scoring and Surgical Factors

During surgery, different factors can lead to different surgical outcomes. For example, a longer operation time may increase the chance of infection in the body and damage the peripheral nerves during the operation.

According to the data in Table 3, in this experiment, patients were divided into groups according to the complexity of the surgery, the first group was low-complexity surgery, the second group was medium-complexity surgery, and the third group was high-complexity surgery. According to statistics, the average ischemia time of the first group of patients was 20 minutes, the change in creatinine was about 7%, the average blood loss was 135 ml, and the operation time was 125 minutes. The average ischemic time of the second group of patients was 23 minutes, the change in creatinine was about 15%, the average blood loss was 200 ml, and the operation time was 180 minutes. The average ischemic time of the third group of patients was 35 min, the creatinine change was about 22%, the average blood loss was 220 ml, and the operation time was 230 min. According to this data, the operation time increases as the difficulty of the operation increases.

### 4.3. Imaging-Related Indicators

According to the data in Table 4, the abduction angle of the first group is 41°, the proportion in the safe area is 85%, the anteversion angle is 22°, and the proportion in the safe area is 76%. The second group had an abduction angle of 38°, 90% in the safe zone, and an anteversion angle of 18°, which was 88% in the safe zone. The third group had an abduction angle of 42°, 88% in the safe zone, and an anteversion angle of 17°, which was 87% in the safe zone. The fourth group had an abduction angle of 39°, 89% in the safe zone, and an anteversion angle of 19°, which was 89% in the safe zone.

## 5. Exploration and Analysis of the Selection of T1 Stage Renal Tumor Resection Based on Imaging MAP Score under Smart Medical Care

### 5.1. Image Performance Analysis

With the continuous development of imaging technology, medical imaging examination has become an indispensable inspection method in hospitals, providing strong support for clinical diagnosis.

According to the data in Figure 7, this experiment retrieves the validity of medical images. When the usage rate of Fc1 was 22%, the image efficiency rate was 70%, and when the usage rate was 25%, the image efficiency rate was 69%. When the usage rate is 28%, the image efficiency rate is 68%, and when the usage rate is 31%, the image efficiency rate is 67.3%. When the usage rate was 34%, the image efficiency rate was 67%; when the usage rate was 37%, the image efficiency rate was 60%; when the Fc2 usage rate was 22%, the image efficiency rate was 68%. When the usage rate is 25%, the image efficiency rate is 68.3%, when the usage rate is 28%, the image efficiency rate is 68.1%, and when the usage rate is 31%, the image efficiency rate is 67%. When the usage rate is 34%, the image efficiency rate is 66.5%, and when the usage rate is 37%, the image efficiency rate is 60%. According to this data, there is no significant difference in the imaging efficiency between Fc1 and Fc2.

When the usage rate of Fc3 was 22%, the imaging efficiency rate was 68%, when the usage rate was 25%, the imaging efficiency rate was 65.7%, and when the usage rate was 28%, the imaging efficiency rate was 65.6%. When the usage rate is 31%, the image efficiency rate is 65%. When the usage rate is 34%, the image efficiency rate is 64.5%, and when the usage rate is 37%, the image efficiency rate is 64.1%. When the combined use rate of Fc1 and Fc3 was 22%, the imaging efficiency rate was 73%, and when the utilization rate was 25%, the imaging efficiency rate was 74.6%. When the usage rate is 28%, the image efficiency rate is 72%, and when the usage rate is 31%, the image efficiency rate is 71%. When the usage rate is 34%, the image efficiency rate is 70.7%, and when the usage rate is 37%, the image efficiency rate is 68.3%. According to this data, when Fc1 and Fc3 are used in combination, the imaging efficiency is greatly improved.

Insulin is a protein hormone present in the human body, which can participate in the regulation of glucose metabolism and control the balance of blood sugar. If there is an excess of insulin, it will cause hypoglycemia, which has important effects on the human nervous system.

According to the data in Figure 8, in order to explore the surgical method of renal tumor resection, the experimental group and the control group were set for comparison. According to the left insulin function evaluation data in Figure 8, it can be seen that the insulin function of the control group as a whole showed a trend of first rising and then falling. Insulin function began to recover on the first day after the operation, and the recovery effect was very slow at first, but there would be a sharp rise in the A2 time period and peaked at the A3 time point. After the A3 time period, the insulin function will show a downward trend, and the downward trend is relatively large at first. After the A4 time period, the decrease in insulin function will become smaller and gradually maintain a stable state. The insulin function data of the experimental group showed that on the whole, the rise and fall time points of insulin function were similar to those of the control group. However, there is a big difference in the specific values, and there is no significant difference between the experimental group and the control group in the initial value. However, in the A2 period, the insulin function of the experimental group far exceeded the normal level and maintained a significant upward trend. The insulin level of the experimental group reached its peak in the A3 period, and the insulin level at this moment was much higher than the normal level, which had a great impact on the postoperative recovery of the patient. Although the insulin function of the experimental group showed a downward trend after the A3 time period, it was still much higher than the normal level. According to this data, the insulin function after renal tumor resection is the object that needs to be paid more attention to.

### 5.2. Complications

In order to verify the effect of the combination of smart medicine and imaging technology in renal tumor resection, we used a method to compare with traditional surgical methods for analysis. The specific conditions are as follows.

According to the data in Figure 9, when using smart medical and imaging technology for surgery, 4 patients, accounting for 11%, developed nausea. There were 3 people with vomiting symptoms, accounting for 8%; 4 people had abdominal distension symptoms, accounting for 11%; 1 person had symptoms of incision infection, accounting for 2.1%; 2 people had symptoms of intra-abdominal bleeding, accounting for 4.2%. There was 1 person with symptoms of urinary tract infection, accounting for 2.1%; there were 2 people with symptoms of ascites, accounting for 4.2%. According to this data, the probability of complications caused by the use of smart medical and imaging technology in surgery decreases. The highest proportion is abdominal distension, and the lowest proportion is incision infection and intra-abdominal hemorrhage.

When the traditional method was used for surgery, 10 patients had nausea, accounting for 24%; 6 patients had vomiting, accounting for 16%; 15 patients had abdominal distension, accounting for 30%; 4 people had symptoms of incision infection, accounting for 10%; 7 people had symptoms of intra-abdominal bleeding, accounting for 18%; 5 people had symptoms of urinary tract infection, accounting for 14%; 6 people had symptoms of ascites, accounting for 16%. According to the comparison between smart medical treatment and imaging technology and traditional methods, there are many complications caused by traditional surgical methods, of which the largest proportion is incision infection and nausea. However, the combination of smart medical care and imaging technology can effectively reduce this situation and reduce the probability of complications as a whole.

### 5.3. Hemoglobin and Creatinine

Hemoglobin is a special protein contained in red blood cells, which has the function of transporting oxygen and plays an important role in the normal physiological functions of the human body. Creatinine is a product of muscle metabolism in the human body and is excreted through the glomerulus.

According to the data in Figure 10, the preoperative hemoglobin in the control group was stable at 130 g/L, and the postoperative hemoglobin was stable at 140 g/L; the preoperative creatinine was stable at 84 mol/L, and the postoperative creatinine was stable at 71 mol/L. In the experimental group, the preoperative hemoglobin was stable at 131 g/L, and the postoperative hemoglobin was stable at 138 g/L; the preoperative creatinine was stable at 84 mol/L, and the postoperative creatinine was stable at 75 mol/L. According to the data, there is no significant difference in hemoglobin between different renal tumor resections, but the recovery of creatinine in the experimental group is better, which shows that the combination of smart medical and imaging technology is beneficial to the postoperative recovery of patients undergoing renal tumor resection.

## 6. Conclusions

With the continuous progress of science and technology, the combination of science and technology and medical treatment has become the general trend. The renal tumor is a common disease nowadays, with a large number of patients, but the investigation found that the complications caused by renal tumor resection are relatively common. The purpose of this paper is to study the research on the selection of T1 stage renal tumor resection based on the imaging MAP score under smart medical care; it is expected to provide help for renal tumor resection through smart medicine and medical imaging technology and to provide new ideas for renal tumor resection. The main work completed in this paper is as follows. (1) Through the comparison of hemoglobin and creatinine content under different surgical methods, it is found that the combination of smart medical treatment and imaging technology is beneficial to the postoperative recovery of patients undergoing renal tumor resection. (2) The combination of smart medical treatment and imaging technology can reduce the probability of postoperative complications. Although this paper has carried out some research on this basis, there are still many problems. (1) The experimental data in this paper are relatively concentrated, which may not represent the general situation and have limitations to a certain extent. (2) There is not much research on the postoperative complications of patients undergoing renal tumor resection, and only simple statistics are carried out.

## Figures and Tables

**Figure 1:** Structure of the intelligent medical system.

**Figure 2:** The original smart medical structure.

**Figure 3:** Detection alert system.

**Figure 4:** Intelligent system diagram.

**Figure 5:** Curve evolution direction.

**Figure 6:** Schematic diagram of the evolution of the horizontal set curve.

**Figure 7:** Image performance analysis.

**Figure 8:** Functional evaluation and thromboplastin analysis.

**Figure 9:** Investigation of postoperative complications.

**Figure 10:** Hemoglobin and creatinine analysis.

**Table 1:** Age distribution of patients.

Age (years)	Male	Ratio (%)	Female	Ratio (%)
0–20	2	1.3	1	0.7
21–40	17	11.4	13	8.8
41–60	25	16.9	19	12.9
60–80	39	26.6	32	21.7
Total	83	56.1	65	43.9

**Table 2:** Scoring and surgical approach.

Group	Number	Surgical approach		
		Open	Laparoscopy	Simple laparoscopy	Imaging laparoscopy
1	19	9	20	7	13
2	60	25	35	25	10
3	40	32	8	5	3

**Table 3:** Analysis of the correlation between scores and surgical factors.

	1	2	3
Ischemia time (min)	20	23	35
Creatinine change (%)	7	15	22
Volume of blood loss (ml)	135	200	220
Time (min)	125	180	230

**Table 4:** Imaging-related indicators.

Group	1	2	3	4
Number	65	60	80	70
Angle of abduction (°)	41	38	42	39
Proportion (%)	85	90	88	89
Anteversion angle (°)	22	18	17	19
Proportion (%)	76	88	87	89

## Data Availability

No data were used to support this study.
